# IGBT Fault Prediction Combining Terminal Characteristics and Artificial Intelligence Neural Network

**DOI:** 10.1155/2022/7459354

**Published:** 2022-07-14

**Authors:** Cailin Li

**Affiliations:** ^1^School of Architecture and Transportation Engineering, Guilin University of Electronic Technology, Guangxi, China; ^2^Guangxi Key Laboratory of Manufacturing System & Advanced Manufacturing Technology, School of Mechanical and Electrical Engineering, Guilin University of Electronic Technology, China

## Abstract

The insulated gate bipolar transistor (IGBT) is widely utilized in the transportation, power, and energy domains because of its high input impedance and minimal on-voltage drop. IGBTs are frequently used in industrial applications for lengthy periods of time, collecting fatigue damage and eventually aging and failing, which can result in system shutdown and financial losses in severe circumstances. As a result, a study into the IGBT's reliability is extremely important. Fault prediction technology, which is an important aspect of reliability research, may analyze device state through changes in terminal parameters, anticipate aging trends, and issue early warnings at thresholds to avoid significant safety issues caused by IGBT aging failures. Therefore, the appropriate end parameters are selected as aging characteristic parameters, and fault prediction is performed. Therefore, this paper has carried out research on the IGBT fault prediction technology that integrates the terminal characteristics and artificial intelligence neural network. The main research contents include the following: (1) this paper starts from the basic principle of IGBT and the structure of its device and analyzes its failure mode on the failure of IGBT. The characteristic parameter of collector-emitter turn-off peak voltage value is selected for IGBT fault prediction, and the aging data of NASA PCoE Research Center is used to verify that the characteristic parameter can be used for fault prediction. (2) In view of the shortcomings of traditional fault forecasting methods, this paper proposes to use deep learning time series forecasting methods for fault forecasting. The LSTM is theoretically analyzed, and the prediction network is built. The experimental results show that the LSTM network model can improve the accuracy of IGBT fault prediction, with fewer parameters and higher prediction efficiency.

## 1. Introduction

As the most important component in a power electronic system, IGBT is the first-choice module for power semiconductor devices. IGBT was invented in 1982. Although it is a very new type of power semiconductor device, it is still developing and improving. From the point of view of power consumption, when the rated current of the IGBT is 75 A and the rated voltage is 600 V, the rated power of the first generation IGBT is 100 watts, and now, it is less than 30 watts. At present, the maximum collector current of the IGBT has been more than 3500 A [1]. From the point of view of the manufacturing process, the current IGBT process is already less than 1 micron. At the same time, the gate trenching technology is adopted in the fourth-generation products, and the size of the chip is also reduced by 80% compared with the previous generation [2]. With the continuous improvement and optimization of the performance and volume of IGBTs, it is reasonable to seize most of the power electronic equipment market. Its superior performance and low power consumption are powerful tools to promote the development of the new energy era. At present, the application prospect is very broad, and it is an indispensable part of many fields such as rail transit, household appliances, infrastructure, and new energy vehicles. For example, in the “heart” of the train, the traction converter uses IGBT modules [3]. The above are all civil fields. For other fields such as aerospace equipment, IGBT also plays a key role. It can be said that the status of IGBTs for power electronic systems is not lower than that of CPUs for computer systems. IGBT modules, on the other hand, have a very high internal resistance under high pressure or high temperature, are prone to high conduction loss, and are not very resistant to high impact force, so they are used in harsh production environments, or after long-term use, they will gradually age or even fail, causing the equipment to stop running, and even the entire power system to be paralysed, causing serious economic losses and even threatening human life [4]. According to the statistics of the British Wind Energy Agency, before 2009, more than 700 wind turbines were burned in the world, many of which were caused by the failure of IGBTs. The reliability of IGBTs plays an important role in the smooth operation of power electronic systems, so it is very meaningful to study the causes of IGBT failures and fault prediction [5]. Before IGBT failure prediction, it is necessary to first study the cause of IGBT failure, that is, the failure mechanism of IGBT. After understanding the changing trend of the degradation parameters before the IGBT fails, measure these parameters. When the parameters are found to be abnormal or about to reach the alarm threshold, it means that the device may fail, so that it can be repaired or replaced in time to avoid more serious accidents [6]. Not only that, while avoiding equipment failure, it can also automate maintenance and repair, redundant copy replacement, etc., which improves the efficiency and cost of operation management and reduces the burden of manual maintenance. In this context, in order to reduce the heavy losses caused by the shutdown of the power system due to IGBT failure during the operation of power electronic equipment and improve the stability of the power system operation, countries around the world are actively carrying out IGBT fault prediction research [7]. The direction of its fault research can be roughly divided into two types: one is based on the machine model and probability model of IGBT, the focus of the research is mainly on the characteristics and materials of the device itself, and the fault prediction model is obtained through statistical analysis of a large number of aging experimental data. The other is an intelligent algorithm prediction model driven by IGBT data. The focus of the research is on the data drive of degradation parameters. Consider using intelligent algorithms such as popular neural networks to build fault prediction models [8]. In today's intelligent world, the rapid development of ANN has ushered in a data-driven era. Finding the relationship between features and targets through data is the mainstream direction of the current social forecasting development. In this paper, the terminal characteristics and neural network are combined to predict the fault of IGBT, because the neural network has incomparable advantages in dealing with nonlinear problems. It provides a good solution for data prediction of nonlinear, time-varying, strongly constrained, large-lag processes.

The following is the paper's organization paragraph: In Section 2, the related work is provided. The suggested work's methods are examined in Section 3. The experiments and results are discussed in Section 4. Finally, the research job is completed in Section 5.

## 2. Related Word

Abroad, Reference [9] proposes a physical model for life estimation of standard power modules. The proposed model can physically explain the dependence of life on various characteristics of the temperature profile, such as frequency, maximum, and minimum temperature. The model uses the Clech method to simulate the stress-strain solder response under cyclic thermal loading and uses a solder deformation mechanism diagram to describe the dominant failure mechanism under stress-temperature circumstances. Reference [10] studied the fundamental frequency thermal cycle and proposed a life estimation method for modular multilevel converter submodules based on the combination of finite element analysis and physical life model. This method provides a more in-depth physical description of the failure mechanism and takes into account the thermal coupling between chips, making life calculations more accurate. Reference [11] obtained the thermomechanical stress distribution around the IGBT defect through finite element analysis, gave a life model combined with the performance of the solder layer, and then verified the model through power cycling experiments and microscale CT scanning. Reference [12] demonstrated the influence of solder joint thickness on the service life of power semiconductor IGBT, and based on this, the optimization problem of solder layer thickness was studied. In China, Reference [13] considers the failure position of the solder layer and the feedback effect of thermal characteristics caused by fatigue, establishes a multiphysics coupling simulation of IGBT, uses an update strategy based on the Cauer thermal network model, and establishes a method that takes into account the cumulative effect of solder layer fatigue. The IGBT life prediction model of the wind turbine converter is finally evaluated. The analytical life model of IGBT mainly describes the relationship between load current, current frequency, average temperature, temperature fluctuation value, temperature rise rate, and other factors and the number of failures, that is, life. At present, the life model provided by device manufacturers is mainly based on the average temperature. In the relationship between the temperature fluctuation value and the number of failures, the number of failures is obtained by power cycle or temperature cycle experiments. Reference [14] established the finite element model of the IGBT model SKM50GB12T4, considering the influence of the power cycle load temperature level on the fatigue life of the solder layer of the device, improved the Coffin-Manson model, and applied the improved model to the IGBT life prediction. In China, by analyzing the failure mechanism of IGBT, Reference [15] designed a power cycle experiment and formulated an experimental plan, used the Weibull distribution to obtain the parameters of the device life model, and then established the Coffin-Manson-Arrhenius life model. The model has higher accuracy, and the effect of junction temperature is more in line with the actual situation. The fault prediction approach based on terminal characteristics compares characteristic parameters in the actual operating state with known aging characteristic parameters of the device, judges the current operating condition, and predicts future parameter trend curves. When the specified aging threshold is reached, the aging IGBT can be maintained, repaired, or replaced in time. The core of this method is to extract and transform historical data and use some intelligent algorithms to estimate the trend of the device's future operating state. Its key technologies include aging feature parameter extraction and prediction algorithm design, and mainstream algorithms include regression algorithms in numerical algorithms, filtering algorithms, and artificial neural networks (ANNs) in machine learning.

Abroad, a research group from Cranfield University used the collector-emitter voltage *V*_CE_ of IGBT as a characteristic parameter, established a random degradation model based on probability distribution, and studied the effects of the gamma distribution, exponential distribution, Poisson distribution, and combined distribution models on IGBTs. The accuracy of life prediction is improved, and the failure model based on a time-delay neural network (TDNN) is used to improve the prediction accuracy. Compared with the method based on the stochastic model, the error of the prediction method based on TDNN is less than 4% [16–18]. Reference [19] studied the fault prediction framework of IGBT. The framework uses the Mahalanobis distance method for abnormality monitoring. After monitoring the abnormality, the particle filter (PF) method is used to predict the fault time, and the collector-emitter saturation voltage is selected. Decreasing *V*_CE (ON)_ is an aging characteristic parameter, and its value increases by 20% as the failure threshold. The prediction error of the research and analysis algorithm is 20%. Reference [20] studied a fault prediction method based on a neural network and adaptive neurofuzzy inference system and used it to predict the degradation of IGBT devices, using the IGBT collector-emitter voltage degradation life data in the NASA Research Center database to compare the proposed method. For verification, the prediction errors of the two methods are 19% and 31%, respectively. The fault prediction method based on end characteristics does not require the mathematical model and physical model of the object and estimates the future operation trend of the object based on the condition monitoring data, thus avoiding the shortcomings of the model-based fault prediction method, but in practical engineering applications, some historical data are difficult to obtain or expensive to obtain, and the obtained data also has certain uncertainty and incompleteness, which increases the difficulty of the method based on end characteristics [21, 22]. Moreover, the traditional prediction algorithms used in some literature cannot make full use of the historical information of the data, resulting in inaccurate prediction and low precision. Therefore, how to effectively use the time-series information of the data is also an important point. There are many classifications of intelligent algorithms in fault prediction based on terminal characteristics, especially in the field of machine learning led by neural networks, which have unparalleled advantages in solving nonlinear problems, and some of them also have good solutions to time series problems, and more importantly, it is more in line with the current trend of rapid development of big data technology.

## 3. Method

### 3.1. IGBT Aging Characteristic Parameter Selection

The aging failure or failure of IGBT will lead to changes in its physical and chemical properties; that is to say, the aging failure problem of IGBT will be manifested in its terminal parameters to a certain extent. Therefore, on the basis of studying the failure mechanism of IGBT, the terminal parameters that best represent its health state can be selected as the aging characteristic parameters and combined with some intelligent algorithms to predict the failure. This section will list the key terminal parameters of IGBT and analyze the changes in their values with aging and finally select appropriate parameters as aging characteristic parameters. The terminal parameters of IGBT devices mainly include gate turn-on threshold voltage, module thermal resistance value, collector-emitter saturation voltage value, and collector-emitter turn-off peak voltage value. Each eigenvalue is analyzed below.

#### 3.1.1. Gate Turn-On Threshold Voltage

The gate turn-on threshold voltage is the minimum voltage value for the IGBT to ensure that the device can be turned on. As the IGBT gradually degrades and fails, the material layer at its gate will gradually degrade, resulting in a larger turn-on voltage during the turn-on process. This indicates that the gate turn-on threshold voltage gradually increases during the IGBT degradation process, which can be used as a characteristic parameter for fault prediction. However, the gate voltage in a normal application environment is controlled by a steady source circuit signal, and it is difficult to effectively detect the gradually changing minimum turn-on threshold voltage.

#### 3.1.2. Module Thermal Resistance Value

Since the IGBT works in a high-temperature and high-pressure environment for a long time, its degradation effect is very obvious, resulting in expansion cracks in the device material layer, which increases the thermal resistance value of the module and the junction temperature value of the module, further accelerating the degradation of the device. For the detection of junction temperature and thermal resistance, it is currently necessary to go deep into the device for measurement, which can still be achieved in the experimental environment, but it is difficult to effectively measure the IGBT device in normal use, which is not conducive to using this characteristic parameter for IGBT fault prediction.

#### 3.1.3. Collector-Emitter Saturation Voltage Value

The IGBT is in the off-and-on state for a long time, and its ideal equivalent principle can be compared to a lossless on-off switch. However, in practical applications, there will be internal on-off resistance. This results in a voltage drop between collector and emitter. Some literature studies have shown that the voltage between the collector and the emitter is not constant, but changes with the degradation of the IGBT. During the degradation process, the collector-emitter saturation voltage value is gradually rising, so it can be a characteristic parameter for IGBT fault prediction.

#### 3.1.4. Collector-Emitter Turn-Off Peak Voltage Value

During the IGBT turn-off process, due to the existence of the parasitic transistor, the transistor generates a transient voltage, and this voltage and the IGBT collector-emitter voltage work together to generate an instantaneous peak voltage. At the moment of a turn-off, the *V*_CE_ of the IGBT will have a high peak value, the turn-off current will drop rapidly, and the turn-off voltage will rise rapidly. When the voltage rises, there will be a voltage value exceeding the normal voltage, and there will be a protruding peak in the waveform. The existence of this overvoltage will cause stress shock to the device, so it is very necessary to analyze the voltage value. Analysis of laboratory aging data shows that when the IGBT degradation changes, the instantaneous peak voltage of its turn-off is gradually decreasing, so this parameter can be used to predict IGBT faults.

Through the comparison of experimental data, the collector-emitter turn-off peak voltage value shows a downward trend in the process of IGBT degradation, and the effect is obvious, while the collector-emitter saturation voltage value has no obvious upward trend in this data set. From the previous theoretical analysis and degradation experimental data, it is shown that the collector-emitter turn-off peak voltage value can be well used as the characteristic parameter of IGBT fault prediction. This paper will select this characteristic parameter and use this data set to study the IGBT fault prediction algorithm. Write a Python program to extract the peak voltage value of each group of data and obtain a total of 540 groups of peak voltage values.

### 3.2. Time Series Forecasting Methods

The purpose of failure prediction is to find out the failure of the device in advance so that the staff can deal with it in time and reduce the loss of system operation. The traditional IGBT fault prediction method is to use mathematical statistics to mathematically model the IGBT degradation parameters, but this method fails to make full use of the data time series information, and the model is difficult to apply to complex production and life. Machine learning algorithms and BP neural network algorithms have significantly improved prediction accuracy. However, the IGBT failure process gradually degrades with time. Therefore, this paper focuses on the application of deep learning time series prediction algorithms in IGBT fault prediction. The time series forecasting method developed earlier, there are many forecasting methods, and the application is also very wide. The traditional time series forecasting method is developed from the mathematical statistics theory, and now, there are many branches of forecasting methods. The nature of prediction can be divided into quantitative analysis method and qualitative analysis method, and many subsequent prediction methods are also evolved on the basis of this method. The regression methods such as univariate linear regression evolved from the causal prediction method to determine the relationship between data samples by means of data processing. In the process of modeling regression, this method does not make full use of the contextual relationship of the data sequence, and it is difficult for the regression model to make effective predictions on future data. The moving average method evolved from the trend forecasting method uses time-series historical information for forecasting. The moving average method mainly seeks the average value of a historical time series for a stationary time series to predict the data. The weighted moving method is an improvement and improvement of the moving average method. It mainly weights the historical information, assigns different weights to different historical information, and then predicts the future data. The moving average method has good prediction accuracy for stable series, but it is difficult to apply effectively to nonstationary series. The weighted movement method needs to retain the information of the entire historical sequence when forecasting, and its forecasting efficiency is greatly reduced in the face of the huge amount of data forecasting.

With the continuous progress of science and technology in recent years, AI has developed rapidly. The model function fitting ability of AI algorithms is much higher than that of traditional modeling methods.

#### 3.2.1. Decision Tree

It is a method of using information gain to predict or classify data, and its commonly used forms are decision trees such as ID3 and C4.5. This method realizes the decision-making model through continuous attribute judgment and decision-making and achieves the application purpose. However, when constructing the model, the decision tree ignores the relationship between attributes and features, and it is more prone to decision bias for data with unbalanced samples.

#### 3.2.2. Bayesian Network

It is a directed acyclic graph model, which represents a set of conditional probabilities, and can also be regarded as a nonlinear extension of a Markov chain. The advantage of this network is that the attribute variables can be connected to make inferences and predictions; the disadvantage is that the training of the network structure is more complicated, and it is not easy to train the model application.

#### 3.2.3. Support Vector Machine (SVM)

SVM is used on various occasions due to its extremely robust performance. It works by efficiently dividing the data by finding the hyperplane with the largest spacing of the data. Support vector regression is to make all the data of a set have the closest distance to the plane, so as to achieve the purpose of data prediction. However, this method cannot fully utilize the historical information of time series.

#### 3.2.4. Neural Network

Due to the strong function fitting ability of neural networks and model construction through learning and training, the application of neural networks has developed rapidly in recent years. Now, the neural network has developed many branches, including back propagation neural network (BPNN), recurrent neural network (RNN), and convolutional neural network (CNN), which are the development and application neural networks. BPNN can fit any nonlinear function, and its prediction model has a strong expressive ability. Due to the influence of its own structure, the RNN has a more obvious solution to dealing with time series problems, such as speech recognition and machine translation. Recent studies have shown that CNN can also perform time series prediction. The method is to use the network to make predictions on the time series data by constructing spatial data information from the sample data time series. To sum up, the time series forecasting method is developing in the direction of AI. Among them, the neural network has been paid more and more attention by scholars and research institutions from all walks of life due to its strong model construction and expression ability.

### 3.3. Deep Learning-Related Technologies

#### 3.3.1. Deep Learning Concepts

The performance and generalization ability of the shallow network model is limited. In order to improve the performance of the model, the artificial neural network (ANN) has been improved and extended. The multilayer and various neural networks are connected and combined, and the training optimization algorithm is improved to construct a network model belonging to the deep neural network (DNN) model. Compared with the shallow network, the improved multilayer network has greatly improved the ability to solve complex problems. Due to the different structures of the neural network, the deep learning neural network includes the following three network structures:

*(1) DNN Network Is Composed of Multilayer Neural Networks*. Compared with the BPNN, it has more layers in general. The complexity of the network model is improved by increasing the number of hidden layers of the network, which is mainly used to solve application problems such as nonlinearity or linearity.

*(2) CNN Is Different from the Fully Connected Network*. It belongs to the partially connected network model. Network layers are connected by convolution kernel operations. This kind of network mainly performs feature processing on images through convolution operations and is mainly used in image processing.

*(3) RNN Is a Network with a Feedback Connection*. Due to the special structure of the network itself, the network has an excellent effect in dealing with time series problems, mainly used for speech recognition and time series prediction. RNN has developed rapidly in recent years, and a variety of improved RNN structures have been formed, such as the Long Short-Term Memory Network (LSTM) structure and GRU structure. In the application, in order to improve the use effect, most of them use a combination of various network structures to improve the performance of the model. In this paper, RNN such as LSTM is used in the study of IGBT fault prediction. And use the combined network model to improve the prediction network, and finally explore the best prediction network, model.

#### 3.3.2. Loss Function

Compared with the actual value, the predicted value obtained by the neural network model will have a certain error. During the model training process, we always hope that the error value can gradually become smaller. The function that measures the error distance between the predicted value and the true value is called the loss function. The loss function is used to update the weights during training so that the loss function is gradually reduced and the model parameters are continuously optimized. The selection of the loss function is related to the occasion to be applied. Common loss functions include cross-entropy, maximum likelihood error, maximum a posteriori probability, and mean square error. This paper studies the IGBT fault prediction problem, and the prediction problem belongs to the regression problem. Formula (1) shows the expression of the mean square error loss function:

(1) $$\begin{array}{c} L_{\left(\sigma \right)}=\frac{1}{n}\overset{n}{\underset{i=1}{\sum }}{\left(y^{i}-y_{\sigma }\left(x^{i}\right)\right)}^{2}, \end{array}$$

where *L*_(*σ*)_ represents the error between the real value and the predicted value, that is, the loss function; *n* is the number of training samples; *y*^*i*^ represents the real value; *σ* is the parameter variable of the network; and *y*_*σ*_(*x*^*i*^) represents the predicted value of the network model. The larger the value of *L*, the greater the deviation between the predicted value of the network model and the true value. The process of deep learning network training is to continuously fit the prediction function model by continuously reducing the loss function value.

### 3.4. IGBT Fault Prediction Based on LSTM

#### 3.4.1. LSTM Network

Due to the existence of the cyclic structure of the RNN network introduced above, when using the chain derivation rule for gradient descent, it is very likely that the gradient disappears or the gradient explodes. Therefore, the long-term dependence of the RNN network makes it difficult to apply for a long-time sequence. In order to solve the impact of a long-term dependence on RNN, the long-short-term memory network LSTM came into being. LSTM is a special loop structure that learns information in network parameters through the control of three gate structures. The LSTM structure has three “gates,” namely, the input gate, forget gate, and output gate. The calculation method of the LSTM unit is shown in the following formulas:

(2) $$\begin{array}{c} f_{t}=\mu \left(W_{f}^{T}\times h_{t-1}+U_{f}^{T}\times x_{t}+d_{f}\right),\\ i_{t}=\mu \left(W_{i}^{T}\times h_{t-1}+U_{i}^{T}\times x_{t}+d_{i}\right),\\ C_{t}^{\prime }=\tanh\left(W_{C}^{T}\times h_{t-1}+U_{C}^{T}\times x_{t}+d_{C}\right),\\ O_{t}=\mu \left(W_{O}^{T}\times h_{t-1}+U_{O}^{T}\times x_{t}+d_{O}\right), \end{array}$$

where *W* and *U* represent the weight parameters of the corresponding gate structure.

#### 3.4.2. LSTM Prediction Network Design

From the analysis of the LSTM network structure in the previous chapters, we can see that the special structure of the LSTM network makes it possible to solve time series problems. The special gate structure of LSTM can store input information of longer time series and prevent the problem of gradient disappearance. The advantages of LSTM are as follows:

1. It solves the long-term dependence problem of RNN, enabling it to learn information from long time series
2. LSTM network has strong data fitting ability, and its robustness and versatility are strong
3. The network parameters of the recurrent layer are shared, and their parameters do not increase with the length of the time series. Due to the special structure of LSTM and its advantages for time series processing, the LSTM network can be used for IGBT fault prediction tasks. Next, a prediction network will be designed step by step for the IGBT fault prediction problem

*(1) The Input and Output of the Network*. The input of the LSTM network is time-series data, and its sequence length can be set to *T*. For the network output part, LSTM has two output forms: one is that the input time series *X*_*T*_ is processed by the network to output the same length of time series data  *Y*_*T*_; the other is that the output contains only one output result value. The input and output of its single-layer LSTM network are shown in Figure 1.

Here, *X*_*T*_ represents a certain sample sequence; *Y*_*T*_ represents the output result sequence, and the following formulas can be used.

(3) $$\begin{array}{c} X_{T}=\left[x_{0},x_{1},\cdots ,x_{t}\right],\\ Y_{T}=\left[y_{0},y_{1},\cdots ,y_{t}\right]. \end{array}$$

Figure 1 shows the two output modes of the LSTM network, which are used in the combination of multi-layer LSTM networks (Figure 1(a)) to pass the time series backward.  Figure 1(b) can be used to get the results when doing the output of a single-layer network or the last layer of a multilayer network.

*(2) Selection of Activation Function*. Sigmoid and tanh activation functions have gradient disappearance in the value range, so the IGBT fault prediction network in this paper will use the Leaky ReLU activation function with better performance to reduce the possibility of gradient disappearance in a recurrent network.

*(3) Hidden Layer Design*. The number of hidden layers and nodes in the hidden layer has an important influence on the output results of the prediction network. The increase in the number of layers and nodes will make the network model more complex and deeper, which will help improve the data fitting ability but is not conducive to network training. There is no specific theoretical basis for the design of the hidden layer, and it is generally set according to an empirical formula. When setting, you can refer to the empirical formula such as

(4) $$\begin{array}{c} h=\sqrt{m+n}+b, \end{array}$$

where *h* is the number of hidden layer nodes, *m* is the number of input layer nodes, *n* is the number of output layer nodes, and *b* is a constant value of about 10.

*(4) Loss Function*. This paper studies the problem of IGBT fault prediction, so the mean square error is chosen as the loss function of the network.

*(5) Prevent Overfitting Method*. Overfitting means that the trained network model performs well in the training set, but the performance in the test set is poor, making it difficult to apply in practice. Since the network model has many parameters and is prone to overfitting, it is necessary to optimize the model by limiting overfitting. Commonly used methods to limit overfitting include *L*_1_ and *L*_2_ regularization, both of which are optimized by “penalizing” weight parameters. Formulas (5) and (6) show the calculation methods of these two regularization methods:

(5) $$\begin{array}{c} L_{1}=L_{\left(\sigma_{n}\right)}+\lambda \overset{n}{\underset{i}{\sum }}\left|\sigma_{i}\right|, \end{array}$$

(6) $$\begin{array}{c} L_{2}=L_{\left(\sigma_{n}\right)}+\lambda \overset{n}{\underset{i}{\sum }}\sigma_{i}^{2}, \end{array}$$

where *L*_(*σ*_*n*_)_ represents the loss function and *λ* represents the regularization coefficient, which is generally set to 0.5. Since *L*_1_ regularization produces sparse solutions, this paper uses the *L*_2_ regularization method to prevent overfitting when designing an IGBT fault prediction network.

In this paper, the IGBT fault prediction network will use the above design method to design the prediction network and explore the best IGBT fault prediction network model by changing the LSTM network with different hidden layers, different nodes, and different time series lengths.

### 3.5. Predictive Evaluation Indicators

In order to facilitate the comparison of the prediction effect of the prediction method network, it is necessary to quantify the prediction results to measure the quality of the prediction results of the network model. Evaluation indicators need to be appropriately selected according to actual problems. The IGBT fault prediction problem studied in this paper belongs to regression analysis, so the regression prediction index can be used to evaluate the model effect. In this paper, the following two regression prediction evaluations are finally selected.

#### 3.5.1. Mean Absolute Error (MAE)

MAE reflects the mean absolute difference between the predicted value and the true value, and its calculation formula is shown in

(7) $$\begin{array}{c} \text{MAE}=\frac{1}{n}\overset{n}{\underset{i=1}{\sum }}\left|y-\hat{y}\right|, \end{array}$$

where *y* represents the real value, $\hat{y}$ represents the predicted value, and *n* represents the number of predicted samples.

#### 3.5.2. Root Mean Square Error (RMSE)

The definition of RMSE is shown in

(8) $$\begin{array}{c} \text{RMSE}=\sqrt{\frac{1}{n}\overset{n}{\underset{i=1}{\sum }}{\left(y-\overset{\wedge }{y}\right)}^{2}}, \end{array}$$

where *y* represents the real value, $\hat{y}$ represents the predicted value, and *n* represents the number of predicted samples.

## 4. Experiment and Analysis

### 4.1. Data Normalization

For network training, data samples are essential. The dimensions of the samples in the original data are different, and the value ranges are inconsistent, which could lead to bias in the network prediction outputs due to the values of different attribute values in the network training. The network is likely to ignore a little value, impacting network training, and prediction accuracy. The scaling of data so that it falls inside a tiny defined interval is known as data normalization. Standardizing the data reduces the impact of varied dimensions and values on network training, improves prediction accuracy, and places the data in the gradient-sensitive part of the activation function, which speeds up network training. In this paper, the following normalization methods are used for data normalization in fault prediction data processing, and its data is normalized to between [0, 1] according to the most typical normalization range.

(9) $$\begin{array}{c} \delta_{i}=\frac{x_{i}-X.\text{Min}}{X.\text{Max}-X.\text{Min}},\\ {\hat{x}}_{i}=\frac{\delta_{i}}{\text{Max}-\text{Min}}+\text{Min}, \end{array}$$

where *x*_*i*_ represents the sample value, *X*.Min represents the minimum value in the sample, *X*.Max represents the maximum value in the sample, Min represents the minimum value of the specified scaling, Max represents the maximum value of the specified scaling, and ${\hat{x}}_{i}$ represents the value after normalization.

### 4.2. Sliding Time Window Samples

Failure prediction methods have been described in previous chapters, and LSTM networks are capable of processing time series data. The input data of the LSTM network are time-series samples, so it is necessary to construct time series samples when training the network and predicting the output. The NASA PCoE dataset used in this paper to study IGBT fault prediction contains 540 collector-emitter turn-off spike voltage values. Because spike voltage values are discrete data values, autocorrelation time series data samples for input to the LSTM network must be created. The sliding time window method is used in this paper to create data samples for network training. The sliding time window method moves on the data value using the supplied input sequence length as the size of the sliding window, uses the value following the window sequence as the sample label value, and generates data samples for training while sliding. The process of the sliding window method is shown in Figure 2.

Among them, the Figure 2 shows the construction process of time series data samples with a sequence length of 5 by the sliding window method. For example, [[*x*0, *x*1, *x*2, *x*3, *x*4], [*x*5]] represents a time series sample constructed by the sliding window method, and [*x*5] represents the sample label value. This paper uses the sliding window method when constructing time-series samples and uses the previous time series values to predict the next sample point. First, write a Python program to normalize the 540 values of NASA PCoE data using the data normalization method in the previous section, and write a function program for constructing time series samples in Python to construct time series lengths sample sets of 5, 10, 15, 20, and 25, and use 80% of the time series samples for training and 20% for testing.

### 4.3. LSTM Network Experimental Results and Analysis

This section conducts IGBT fault prediction experiments based on the LSTM network. Set different time series lengths, different network layers, and different hidden layer nodes to explore the best fault prediction model of LSTM. In the LSTM network experiment, the learning rate is set to 0.001; the LSTM network layer is set to 1 and 2 layers; the hidden nodes of each layer are set to 30, 40, and 50 nodes according to the empirical formula, and the time series length is set to 5, 10, 15, 20, and 25; batch size is set to 10; adjust each parameter and the number of model iterations to make the model converge to the best. The first 80% of the constructed sample set is utilized for dry training, while the remaining 20% is used for dry testing. Keras is a Python library of deep learning techniques that improves and simplifies TensorFlow. In this paper, Keras and Python are used to create programmer algorithms based on network architecture and to conduct prediction effect experiments. On the IGBT fault curve, LSTM network prediction is conducted using the above parameter settings. To explore the influence of different network depths, nodes, and time series lengths on the prediction results, the single-layer LSTM, 30-node, 40-node, and 50-node network fault prediction experiments are now performed. The experimental results are shown in Table 1 and Figures 3 and 4.

Table 1 and Figures 3 and 4, show the error results of 30, 40, and 50 nodes of a single-layer LSTM network. The normalization (RMSE) in the table represents the root mean square error value of the data value after normalization, 5, 10, 15, 20, 25 indicates the set time series length.

At the same time, this paper also adds a two-layer LSTM network to explore the fault prediction results, as shown in Table 2 and Figures 5 and 6.

Table 2 and Figures 5 and 6 show the error result values of nodes 30, 40, and 50 of the two-layer LSTM network. The normalization (RMSE) in the table represents the root mean square error value of the data values after normalization; 5, 10, 15, 20, and 25 represent the set time series length. When the LSTM network experiment is deepened again, the adjustment parameters cannot converge the model, and the network that is too deep cannot learn the sample data. Therefore, in the above network experiment results, a network model that can predict IGBT faults better is found.

The preceding experimental findings show that correctly expanding the length of the time series can increase the network model's prediction accuracy. When the time series is changed from 5 to 20, for example, the MAE decreases. Similar to single-layer LSTM, when the number of LSTM network layers is raised, the MAE and RMSE in 15 and 20-time series have lower error values, and the prediction model's accuracy improves. After the above experimental results, it is found that when the network parameters are set to the LSTM layer number of 2, 50 nodes, and the time series of 20, the RMSE and MAE error values for IGBT fault prediction are the smallest.

## 5. Conclusion

With the advancement of science and technology, the use of power electronic gadgets has increased dramatically. IGBTs are being used with increasingly powerful system equipment. Furthermore, IGBT devices offer numerous advantages, resulting in an increase in the use of IGBTs and an increase in the number of applications. However, due to the hostile working environment and high working intensity of the IGBT during usage, the IGBT suffers significant fatigue damage, increasing the likelihood of failure. The majority of traditional IGBT fault prediction research relies on fault characteristic parameters for mathematical statistics or uses machine learning methods to construct prediction models. These models fail to make full use of the historical damage information in the process of IGBT degradation over time, and the prediction accuracy is not high. It is difficult to combine with practical application. This article has read a large number of IGBT fault research papers and deep learning algorithm prediction data and has a deep understanding of the current IGBT fault prediction. In this paper, a fusion of terminal characteristics and a deep learning time series prediction algorithm is proposed to predict the fault of IGBT, and the fault prediction network is designed according to the theoretical analysis and experimental results, and the optimal IGBT fault prediction LSTM network model is finally obtained. The main research work in this paper is as follows: (1) This paper starts from the basic principle of IGBT and the structure of its device and analyzes its failure mode on the failure of IGBT. The characteristic parameter of collector-emitter turn-off peak voltage value is selected for IGBT fault prediction, and the aging data of NASA PCoE Research Center is used to verify that the characteristic parameter can be used for fault prediction. (2) In view of the shortcomings of traditional fault forecasting methods, this paper proposes to use deep learning time series forecasting methods for fault forecasting. The prediction network is developed once the LSTM is theoretically studied. The experimental results suggest that using the LSTM network model, which has fewer parameters and a greater prediction efficiency, can increase the accuracy of IGBT failure prediction.

## Figures and Tables

**Figure 1:** LSTM network output method.

**Figure 2:** Sliding window method.

**Figure 3:** RMSE for different number of nodes in a single-layer LSTM.

**Figure 4:** MAE for different number of nodes in a single-layer LSTM.

**Figure 5:** RMSE for different number of nodes in a two-layer LSTM.

**Figure 6:** MAE for different number of nodes in a two-layer LSTM.

**Table 1:** Normalized RMSE for different number of nodes in a single-layer LSTM.

Number of nodes	5	10	15	20	25
30	0.0113	0.0113	0.0138	0.0118	0.0106
40	0.0125	0.0104	0.0118	0.0103	0.0107
50	0.0119	0.0104	0.0103	0.0108	0.0107

**Table 2:** Normalized RMSE for different number of nodes in a two-layer LSTM.

Number of nodes	5	10	15	20	25
30	0.0113	0.0162	0.0109	0.0110	0.0113
40	0.0135	0.0153	0.0106	0.0111	0.0104
50	0.0127	0.0138	0.0107	0.0103	0.0178

## Data Availability

The datasets used during the current study are available from the corresponding author on reasonable request.
